The article "Comparison of Therapeutic Effects between Pulsed and Continuous Wave 810-nm Wavelength Laser Irradiation for Traumatic Brain Injury in Mice" was published in 2011. Journal: PLoS One.

# Comparison of Therapeutic Effects between Pulsed and Continuous Wave 810-nm Wavelength Laser Irradiation for Traumatic Brain Injury in Mice

**DOI:** 10.1371/journal.pone.0026212

**Published:** 2011-10-18

**Authors:** Takahiro Ando, Weijun Xuan, Tao Xu, Tianhong Dai, Sulbha K. Sharma, Gitika B. Kharkwal, Ying-Ying Huang, Qiuhe Wu, Michael J. Whalen, Shunichi Sato, Minoru Obara, Michael R. Hamblin

**Affiliations:** 1 Wellman Center for Photomedicine, Massachusetts General Hospital, Boston, Massachusetts, United States of America; 2 Department of Electronics and Electrical Engineering, Keio University, Yokohama, Japan; 3 Department of Dermatology, Harvard Medical School, Boston, Massachusetts, United States of America; 4 Department of Otolaryngology, Traditional Chinese Medical University of Guangxi, Nanning, China; 5 Laboratory of Anesthesiology, Shanghai Jiaotong University, Shanghai, China; 6 Aesthetic and Plastic Center, Guangxi Medical University, Nanning, China; 7 Department of Burns and Plastic Surgery, Shandong University, Jinan Central Hospital, Jinan, China; 8 Department of Pediatrics, Massachusetts General Hospital, Boston, Massachusetts, United States of America; 9 Division of Biomedical Information Sciences, National Defense Medical College Research Institute, Tokorozawa, Japan; 10 Harvard-MIT Division of Health Sciences and Technology, Harvard University, Cambridge, Massachusetts, United States of America; Massachusetts General Hospital and Harvard Medical School, United States of America

## Abstract

**Background and Objective:**

Transcranial low-level laser therapy (LLLT) using near-infrared light can efficiently penetrate through the scalp and skull and could allow non-invasive treatment for traumatic brain injury (TBI). In the present study, we compared the therapeutic effect using 810-nm wavelength laser light in continuous and pulsed wave modes in a mouse model of TBI.

**Study Design/Materials and Methods:**

TBI was induced by a controlled cortical-impact device and 4-hours post-TBI 1-group received a sham treatment and 3-groups received a single exposure to transcranial LLLT, either continuous wave or pulsed at 10-Hz or 100-Hz with a 50% duty cycle. An 810-nm Ga-Al-As diode laser delivered a spot with diameter of 1-cm onto the injured head with a power density of 50-mW/cm^2^ for 12-minutes giving a fluence of 36-J/cm^2^. Neurological severity score (NSS) and body weight were measured up to 4 weeks. Mice were sacrificed at 2, 15 and 28 days post-TBI and the lesion size was histologically analyzed. The quantity of ATP production in the brain tissue was determined immediately after laser irradiation. We examined the role of LLLT on the psychological state of the mice at 1 day and 4 weeks after TBI using tail suspension test and forced swim test.

**Results:**

The 810-nm laser pulsed at 10-Hz was the most effective judged by improvement in NSS and body weight although the other laser regimens were also effective. The brain lesion volume of mice treated with 10-Hz pulsed-laser irradiation was significantly lower than control group at 15-days and 4-weeks post-TBI. Moreover, we found an antidepressant effect of LLLT at 4-weeks as shown by forced swim and tail suspension tests.

**Conclusion:**

The therapeutic effect of LLLT for TBI with an 810-nm laser was more effective at 10-Hz pulse frequency than at CW and 100-Hz. This finding may provide a new insight into biological mechanisms of LLLT.

## Introduction

Traumatic brain injury (TBI) and its sequelae affect at least 1.4 million people in the United States with an associated mortality of 50,000 and permanent disability of 90,000 each year [1], [2]. The long-term cognitive, psychosocial and physical deficits that follow TBI, lead to an annual economic burden of about 60 billion dollars [3], [4], [5]. For instance, the most frequent psychiatric manifestation seen following TBI is depression, which may affect one-third or more of patients [6], and these patients usually need a variety of long-term services, including rehabilitative therapies, assistive technologies, and expensive medical equipment. A growing number of studies have been carried out for therapy of TBI, however there is no accepted effective treatment so far and clinical trials of pharmaceuticals have generally failed.

In recent times, low-level laser therapy (LLLT) has been clinically applied for a range of medical indications. One of the areas attracting increasing interest is the use of LLLT to treat neurological diseases such as stroke, neurodegenerative diseases, brain injury, and spinal cord injury [7], [8], [9], [10], [11], [12]. The fact there is no effective drug-based therapies for most of these disorders has encouraged researchers to consider the use of laser treatment. Since near-infrared laser can efficiently penetrate into biological tissue including the central nervous system, producing non-invasive beneficial photobiomodulation effects such as promoting nerve regeneration and increasing ATP synthesis. These effects can be attributed to a photochemical mechanism based on light absorption by mitochondrial chromophores rather than the production of heat [13], [14], [15], [16].

The efficacy of LLLT on TBI has been previously investigated to a limited extent. Oron et al. demonstrated that 808-nm Ga-As laser irradiation for a mouse brain traumatized by a weight-drop device promoted long-term restoration of neurological function [17]. More recently, our studies have shown that both 665-nm and 810-nm laser can significantly improve the neurobehavioral performance of mice after severe TBI, while 980-nm laser did not produce the same positive effect [18]. On the other hand, Lapchak et al. compared the neuroprotective effects of LLLT for ischemic strokes in rabbits using 808-nm continuous wave (CW) and pulsed laser [19], [20]. The study demonstrated both 1000-Hz and 100-Hz pulsed laser produced a similar effect on increase in cortical ATP content superior to CW. Thus, some agreement has emerged on the best wavelengths of laser for treatment of TBI, however the effect of laser pulse frequencies on therapeutic modulation for TBI remains unclear.

In the present study, we compared the therapeutic effect using 810-nm continuous wave and pulsed lasers on the neurological and histological outcome of the traumatized mice.

## Results

### Transmitted Laser Power to the Brain Tissue

The measurement of laser power transmission was performed to assess the extent to which transcutaneous and transcranial 810-nm laser irradiation penetrates to the depth of the brain surface. Figure 1 shows the relationship between incident and transmitted laser power in continuous mode. The transmittances with different frequencies (CW, pulsed wave (PW) 10 Hz and 100 Hz) are summarized in Table 1. These results revealed that the transmitted power did not depend on laser pulse frequency; 15% of the incident laser power was transmitted through skin and 6% of that incident power penetrated through skin and skull combined. In the in vivo experiment the 810-nm laser was applied transcutaneously (1-cm diameter spot), while the hole in the skull under the skin was partially present (4 mm in diameter). Thus, the data showed that approximately 3–7.5 mW/cm^2^ of irradiance would reach the brain if the incident irradiance was 50 mW. The measurement of the temperature increase in the brain tissue revealed that the maximum temperature increase during laser irradiation was less than 1°C.

**Figure 1:** Laser transmission through scalp and skull. Plot of measured incident laser power against measured transmitted laser power in CW mode through mouse scalp and scalp and skull combined. Values are expressed as mean ± S.D; n = 3.

**Table 1:** Transmittance of laser power through ex vivo mouse scalp and skull (average ± SD, n = 3).

Transmittance (%)	CW	PW 10 Hz	PW 100 Hz
Scalp	15.25±1.18	14.30±1.30	14.54±1.78
Scalp and skull	6.26±0.68	5.76±0.75	5.90±0.98

### Improvement of neurological severity score (NSS)

Figure 2A shows the changes of NSS at different post-trauma intervals. The initial severity of injury was similar in the four groups of mice as reflected by the NSS at 1 h post-TBI; 7.70±0.15 in the control, 7.70±0.37 in the CW, 7.70±0.15 in the PW 10 Hz, and 7.50±0.22 in the PW 100 Hz (all the groups, *n* = 10). At 48 h after TBI, there was a significant (P<0.01) decrease of NSS in the all three laser treated groups that became even more pronounced (P<0.001) as time progressed and lasted until the end of the study at 28 days. At day 7 it became clear that the improvement in the PW 10 Hz group was greater than that seen in the CW and PW 100 Hz laser treated groups. In order to determine the statistical significance difference between the various laser groups we integrated the NSS for each mouse over the 28-day time course and compared the means of the area under the curve (AUC) values between groups (Figure 2B). The TBI group had a mean AUC that was significantly higher than the treated groups (P<0.0001) and the AUC of the PW 10 Hz group was significantly lower than both the CW group (p = 0,004) and the PW 100 Hz group (P = 0.0018). All groups of mice continued to improve throughout the 28-day duration of the study. The averages of NSS at 4 weeks post-TBI were 2.50±0.27 in the control TBI, 1.30±0.21 in the CW, 0.60±0.22 in the PW 10-Hz, and 1.30±0.26 in the PW 100-Hz laser-treated group, respectively.

**Figure 2:** NSS scores after laser treatment. (A) Time course of neurological severity score (NSS) of mice with TBI receiving either control (no laser-treatment), or 810-nm laser (36 J/cm^2^ delivered at 50 mW/cm^2^ with a spot size of 0.78 cm^2^) in either CW, PW 10 Hz or PW 100 Hz modes. Results are expressed as mean ± S.E.M (n = 10). *** *P*<0.001 vs. the other conditions. (B) Mean areas under the NSS-time curves in the two-dimensional coordinate system over the 28-day study for the 4 groups of mice. Results are means ± SD (n = 10).

### General health and antidepressant effects of laser treatment

Figure 3 shows the changes of body weight measured at different post-TBI time points. As compared with pre-injury levels, body weight was decreased at days 1 and 2 post-injury in the all traumatized mice, while the body weight of the sham-operated mice (just with a craniotomy) was gradually increased. The body weight of laser-treated mice recovered faster and reached a higher level than that of the untreated-TBI mice. The time at which the minimum in the body weight was recorded was 2 days post-TBI in the laser-treated mice (CW; 0.884±0.023, PW 10 Hz; 0.880±0.017, and PW 100 Hz; 0.854±0.024), although untreated TBI mice continued to lose weight up to 5 days post-TBI (0.837±0.043). Body weight almost returned to pre-injury levels at 4 weeks after TBI and tended to continue to increase gradually.

**Figure 3:** Body weight as a measure of health status. Variation of total body weight in healthy (sham control; n = 3), traumatic brain injury (TBI) and 3 groups of 810-nm laser-treated mice (n = 10).

The possible antidepressant effect of LLLT was investigated in the forced swim and tail suspension- behavioral tests. In the forced swim test, there was no significant difference of immobility durations between the groups at 1 day after TBI as shown in Figure 4A. However after 28 days the mice treated with the PW 10-Hz laser showed a significant decrease of immobility time compared to the untreated TBI mice (Fig. 4B). In addition, the immobility periods at 4 weeks post-injury were significantly shorter than those at measured at 1 day after TBI in the all laser-treated groups (CW, PW 10 Hz and 100 Hz), suggesting the antidepressant activity of LLLT. Figure 5 shows the immobility times in the tail suspension test. There was a significant decrease of the immobility periods in the PW 10-Hz laser-treated mice relative to the untreated TBI mice at 1 day post-injury (Fig. 5A). After 28 days, the immobility time significantly decreased in both the PW 10-Hz and the PW 100-Hz laser-treated groups as compared to the untreated TBI mice (*P*<0.01). Moreover, there was a significant difference between the CW and the PW 10-Hz laser-treated mice at 4 weeks post-TBI (*P*<0.05).

**Figure 4:** Forced swim test for depression. Immobility duration in forced swim test (FST) at (A) 1 day and (B) 28 days after brain injury and laser irradiation. Values are in mean ± S.E.M. (n = 10). ‡ *P*<0.05 vs. values at 1 day after TBI. * *P*<0.05 between the groups.

**Figure 5:** Tail suspension test for depression and anxiety. Tail suspension test (TST) showing immobility periods out of 360 sec total test duration carried out at (A) 1 day; and (B) 28 days after TBI and laser irradiation. Values are in mean ± S.E.M. (n = 10). * *P*<0.05.

### ATP contents in the brain after laser

The ATP contents in the traumatized side of the mouse brain were measured immediately after the laser irradiation at 4 h post-TBI to investigate the effect of LLLT on enhancement of mitochondrial function. Figure 6 shows the cortical ATP content in mice brain tissue as a function of treatment groups. For comparison, the ATP content of a normal mouse (not given TBI) was measured. At 4 h post-injury, there was a moderate decrease of ATP content within traumatized cortex as compared to the same cortical region excised from native mice. In the normal mice, baseline cortical ATP content was 21.1±2.9 nmol per mg protein, compared to 15.8±1.1 nmol per mg protein in the untreated TBI mice. The cortical ATP content in the CW and PW 100-Hz mode LLLT treated mice were 18.1±2.1 and 16.1±3.2 nmol per mg protein respectively, while the PW 10-Hz laser treatment resulted in 19.4±3.2 nmol per mg protein. However, the increases were not statistically significantly different from ATP contents measured in the control mice.

**Figure 6:** ATP content in brain. Cortical ATP content in mice brain tissue of left side (traumatic injury) immediately after laser treatment. Values are in mean ± S.E.M. (n = 5).

### Decrease of lesion size in laser treated TBI

The histological assessments of the brain cross-sections removed at 2, 15 and 28 days post-TBI of the untreated TBI mice and the laser-treated mice are shown in Figure 7. Figure 8 shows the quantitative analysis of lesion areas based on the histological images. All mice demonstrated a steady increase in lesion size as time progressed. This is expected as the natural history of TBI is for progressive loss of brain tissue as the lesion progresses [21]. At 15 and 28 days after injury, the untreated TBI mice had a significantly higher loss of cortical brain tissue around the traumatized site compared to the PW 10-Hz laser-treated mice (15 days post-TBI; *P*<0.05, 28 days post-TBI; *P*<0.01). On the other hand, there was no significant difference between the untreated TBI mice and those treated with other modes of laser at any time point. The time course of the progression of cavitary cortical lesions implied a neuroprotective effect of LLLT, particularly at the early stages after TBI.

**Figure 7:** Histology of brain slices. Histological images of cross-sections of brains from control non-laser-treated and laser-treated TBI mice removed at day 28.

**Figure 8:** Area of brain lesions. Results of quantitative analysis of the area of cavitary cortical lesions in brain tissue on the basis of the histological images. Values are means ± S.E.M. (n = 9). * *P*<0.05.

## Discussion

In the present study, we compared the therapeutic effects using an 810-nm diode laser at continuous wave and at two different pulse frequencies as a non-invasive treatment of TBI in mice.

Karu et al. previously suggested that cytochrome c oxidase was a primary photoacceptor when cells are irradiated with far red to near infrared radiation [22]. More recent work has demonstrated that light at both 670-nm and 830-nm can cause the upregulation of cytochrome c oxidase in cultured primary neurons functionally inactivated with potassium cyanide [23]. In other studies, Anders et al. showed that noninvasive transcutaneous application of 810-nm light to spinal cord injury in rats could cause a significant increase in the number of regenerating corticospinal tract axons and the length of axonal regrowth [11], [12]. Our previous report on LLLT for TBI showed that both red laser (665 nm) and near infrared laser (810 nm) can significantly improve the neurobehavioral performance of mice after closed head TBI [18]. Thus, we selected the wavelength of 810 nm in this study to demonstrate the potential therapeutic effect for TBI.

As shown in previous papers, laser power at a wavelength of 810 nm can efficiently penetrate through biological tissue [8], [9], [11], [24], [25]. The most important parameter for the penetration depth of laser in tissue is wavelength, however it is often claimed that a pulsed laser can penetrate more deeply into tissue than CW laser even with the same average power, due to increased penetration of photons at the pulsed peak. Since the peak power is expressed as average power divided by duty cycle, the peak power with a pulsed mode is twice as high as the CW mode in this work (PW; 100 mW/cm^2^, CW; 50 mW/cm^2^). The measurement of the average penetrative power showed the irradiant power to brain tissue was similar regardless of laser frequencies; 15% of the laser power was transmitted through a skin and 6% of that penetrated through a combination of skin and skull. Therefore, the irradiant fluence to a brain was 2.2–5.4 J/cm^2^ since the total fluence for skin was 36 J/cm^2^. The range was consistent with our previous study in where cellular responses of primary cortical neurons to an 810-nm-laser irradiation showed some positive biomodulatory effects such as significant increase of calcium, ATP and mitochondrial membrane potential (MMP) with a laser dose of 3 J/cm^2^ [26]. In addition, the short period of laser irradiation (12 min) was also reasonable in terms of possible clinical application.

The fundamental mechanism of LLLT is proposed to involve photons being absorbed by mitochondria leading to increased cytochrome c oxidase activity [27], release of nitric oxide (NO) [28] and an increase in ATP levels [29], [30]. However, there is a limited attention for the understanding of the pulsing effect on neurological outcome although a recent review did find evidence for the overall increased benefit of pulsed laser over CW laser [31]. The present work demonstrated that the changes of NSS and changes in the antidepressant effect of LLLT were different between the CW, PW 10-Hz and 100-Hz laser irradiation despite the finding that the energy penetrating to the brain was the same.

The efficacy of LLLT for diverse neurological diseases including stroke has been demonstrated in a number of animal and human studies [9], [17], [19], [32], [33], [34] and LLLT also has been shown to improve emotional response and memory performance in middle-aged CD-1 mice [35]. Depression following TBI or stroke is a persistent problem that requires the close attention of medical and rehabilitation professionals [6], [36]. Although, the antidepressant effect of LLLT has not been definitely investigated so far there is one report of transcranial LED (single treatment with 810 nm) improving major depression and anxiety in a 10-patient clinical trial. The results of FST and TST demonstrated that laser irradiation with a pulsed 10-Hz mode efficiently reduced the immobility periods in TBI mice. LLLT could therefore ameliorate a symptom of depression that was possibly a long-term sequela of TBI.

The histological images indicated the prevention of cell death and the protection of neural cells from apoptosis or necrosis at the early stage post-TBI (primary injury) by LLLT. These findings were consistent with some previous reports suggesting LLLT stimulated cell proliferation and inhibited induction of apoptosis [27], [37], [38], while others have shown that too high fluences of light could have deleterious effects on cells by inducing apoptosis via generation of high levels of reactive oxygen species) [39], [40].

Thus, the prevention of neuronal damage would explain the observation that the body weight recovered earlier than the untreated TBI mice and the reduction of cavitary cortical lesions. If the primary injury is severe, it is known that the secondary injury starts to occur about one week after TBI. For instance, some studies showed neurodegeneration after head trauma could be widespread during a period of days to months [41], [42], [43], [44]. Secondary injury results from physiological disturbances caused by the initial damage, and from the development of cerebral ischemia and disruption of the blood-brain barrier [45], [46]. Therefore, the LLLT-induced prevention of cell death at the primary stage could provide the long-term therapeutic effects.

There is some evidence that pulsed light (laser or LED) does have effects that are different from those of continuous mode [31]. Previously, a wound healing study performed by Kymplova et al. concluded a 670-nm laser pulsed at various frequencies (10, 25, and 50 Hz) promoted wound repair more than the CW light source [47]. In research on pain relief, Sushko et al. found that both CW and PW modes of 670-nm laser delivery reduced the behavioral manifestations of somatic pain as compared to the controls, but the application of pulsed light (especially, at 10 and 8000 Hz) was more effective [48]. Moreover, some past studies have shown particular pulsing frequencies appear to be more efficacious than others in triggering desired biological processes [19], [20], [49], [50].

One possible reason why laser irradiation at 10-Hz pulsed mode was most effective for improving neurological outcome is that the hypothesis that the frequency affects the whole brain. Since the brain has waves with specific frequencies, such as alpha waves, beta waves and theta waves, there exists the possibility of resonance occurring between the frequency of the pulsed light and that of the brain waves. Particularly relevant is the fact that oscillation of theta waves that have a prominent 4–10-Hz rhythm in the hippocampal region of all mammals previously studied [51], [52], [53]. The fact that the hippocampus is responsible for behavioral inhibition and attention, spatial memory, and navigation suggests that the significant neurological recovery observed with the PW 10-Hz laser treatment may possibly have resulted from the positive resonance between the pulsing frequency of the laser and the electrical activity of neurons in the hippocampus. In fact, the hippocampus is one of the regions to suffer brain damage in Alzheimer's disease, and a recent study showed that transcranial laser therapy using an 808-nm laser diode attenuated amyloid plaque development in the transgenic mouse model with mutant amyloid- precursor protein, implying the possible efficacy of this therapeutic strategy for Alzheimer's disease [54]. However, further study is necessary to establish whether the resonance effect can explain the superiority of pulsed laser. Another conceivable mechanism for the superiority of pulsed laser over CW is the idea that the pulse duration (100 msec) is similar to some biological time period involved with cell stimulation by laser. This time period could be for instance the half-life of an ion channel in the mitochondrial membrane or some other membrane in the cell that responds to light, one report gave a value of 160 ms [55].

In conclusion, transcranial LLLT with an 810-nm laser improved neurobehavioral recovery in TBI, more effectively at 10-Hz pulsed mode than at CW or 100-Hz pulsed mode. Further studies are necessary to define the detailed mechanisms behind this observation, but the finding may provide novel insight into biological mechanisms of LLLT. Clinical trials of transcranial LLLT for patients who have suffered acute TBI should be considered considering the likely clinical efficacy in stroke and the apparent lack of possible side-effects.

## Materials and Methods

### Ethics statement

All animal experiments were approved by the Subcommittee on Research Animal Care of the Massachusetts General Hospital (protocol number 2009N000006) and were in accordance with the guidelines of the National Institutes of Health (NIH).

### Animal Preparation

Male BALB/c mice (weight 18 to 26 g; Charles River Laboratories, Wilmington, MA) were used in this study. They were housed in groups of 4–5 per cage, in a 12 h: 12 h light: dark cycle. Food and water were provided ad libitem.

### Laser power transmission through skin and skull

Preliminary experiments were carried out with fresh skin and skull removed from sacrificed uninjured mice. Transmission of laser power was determined using a laser power meter capable of measuring pulsed irradiation (Ophir Nova II, North Logan, UT) to measure the transmitted power, and the incident power density using the specified surface irradiance of on the surface of the brain was calculated to be 3–7.5 mW/cm^2^.

### Traumatic Brain Injury Model

Mice were subjected to a single left lateral controlled cortical impact (CCI) with craniotomy [56], [57], [58]. After mice were anesthetized with isoflurane, the top of the skull was exposed with a 1-cm skin incision in the scalp. A craniotomy was performed over the left parietal cortex using a 4-mm trephine attached to an electric drill. The angle of the drill and the head of the mouse were adjusted so that the craniotomy penetrated the thin skull of the mouse without damaging the dura. The 3-mm diameter tip of the impact device (AMS 201, AmScien Instruments, Richmond, VA) was positioned on the left front-parietal cortex and the tip centered 3.0 mm anterior to lambda and 2.5 mm left of midline within the craniotomy. The zero depth position was determined by aligning the tip of the impact device in the down position with the surface of the dura. The depth of injury was set 2 mm using a screw-mounted adjustment. The dwell and total time of the impact device was 50 and 80 msec, respectively. A velocity from 4.2 to 4.9 m/sec was obtained using settings of 150 pounds per square inch (psi) for high pressure and 30 psi for the low pressure when a cylinder of compressed nitrogen (Airgas East, Salem, NH) was connected via a regulator. Immediately after impact the craniotomy hole was sealed with bone wax, the scalp incision was closed with a suture and mice were allowed to recover on a heating pad. At 1 hour post-TBI severity of injury was assessed by neurological severity score (see below). Mice with scores of 7 or 8 were eligible for inclusion in the study, while mice with scores higher or lower that this range were ineligible for inclusion and were sacrificed. A group of control mice (sham-operated mice) received surgery including a craniotomy but no TBI.

### Laser Treatment

Laser treatment was performed 4 h post-TBI using a diode laser of 810-nm wavelength and maximal power output of 3.5 W (DioDent Micro 810, HOYA ConBio, Fremont, CA) equipped with quartz-silica fiber. After mice were positioned on a plastic plate and covered by an aluminum sheet with a 1-cm diameter hole, the distal tip of the fiber optics was set for transcutaneous laser irradiation onto the injured side of the head at a power density of 50 mW/cm^2^. The duration of laser irradiation was 12 min, and the total fluence was 36 J/cm^2^. While the laser mode was set on continuous wave (CW), 10-Hz and 100-Hz pulsed wave (PW) (duty cycle; 50%), the same average power density and total fluence were applied in order to compare the differences of therapeutic effects given by the laser conditions. The complete laser parameters are given in Table 2. Possible heating effect by the laser irradiation was measured by a thermocouple needle-probe of 1.0-mm diameter inserted into the irradiated area in a depth of 3 mm.

**Table 2:** List of laser parameters.

Parameter	Value
Wavelength	810-nm (+/− 2-nm)
Spot size	Diameter = 1 cm, area = 0.78 cm^2^
Average irradiance	50 mW/cm^2^
Total fluence	36 J/cm^2^
Average power	39 mW
Total energy	28 J
Illumination time	12 minutes
A. Pulse frequency	10 Hz
A. Pulse duration	50 msec
A. Peak irradiance	100 mW/cm^2^
B. Pulse frequency	100 Hz
B. Pulse duration	5 msec
B. Peak irradiance	100 mW/cm^2^

### Neurological Severity Score (NSS)

The general health of the mice was monitored for 28 days after injury and the neurological severity score (NSS) was assessed at 1 h, and 1, 2, 3, 5, 7, 10, 14, 21, and 28 days. Body weight was also measured at the same time points. The NSS used in the present study is a modification of the original one reported on the closed-head injury (CHI) model and has been used in a number of studies [59], [60]. The tests are based on the ability of mice to perform 10 different tasks (Table 3) that evaluate the motor ability, balancing, and alertness of the mouse. One point is given for failing to perform each of the tasks, which means a normal and uninjured mouse scores 0, while a score of 10 means likely death.

**Table 3:** Neurological severity score (NSS) for mice.

Neurological Severity Score(NSS) for Brain-Injured Mice	
Presence of mono- or hemiparesis	1
Inability to walk on a 3-cm-wide beam	1
Inability to walk on a 2-cm-wide beam	1
Inability to walk on a 1-cm-wide beam	1
Inability to balance on a 1-cm-wide beam	1
Inability to balance on a round stick (0.5 cm diameter)	1
Failure to exit a 30-cm-diameter circle (for 2 min)	1
Inability to walk straight	1
Loss of startle behavior	1
Loss of seeking behavior	1
Maximum total	10
One point is awarded for failure to perform a task.	

For each failed task the mouse receives 1 point. Maximum = 10 (failure in all tasks), minimum = 0 (success in all tasks).

### Forced Swim Test (FST)

Forced swimming-induced immobility in mice was carried out as described by Porsolt et al. [61], [62] and modified by Aley et al. [63]. Mice were gently placed in a transparent cylinder (20 cm in diameter) filled with water (23–25°C). Filling the cylinder to a depth of 12 cm prevented mice from using their tails to support themselves in water. A mouse was considered as immobile when it remained in an upright position with only minimal paw movements permitted to keep the head above water. Immobility was sampled the predominant behavior over every 5 s during the last 4 min of a 6-min test session [64].

### Tail Suspension Test (TST)

The tail suspension test was conducted as previously described [65], [66]. The method is based on the observation that a mouse suspended by the tail shows alternate periods of agitation and immobility. Mice were securely fastened by the distal end of the tail to a flat stick surface and suspended in a visually isolated. The presence or absence of immobility, defined as the absence of limb movement, was sampled over a 6-min test session.

### ATP Measurement

ATP fluorometric assay kit (K354-100, BioVision, Mountain View, CA) was used according to the manufacturer's instructions to measure the ATP contents in mouse brain immediately after the laser irradiation at 4-h post-TBI. Briefly, brain tissue was homogenized in 1-mL of cell lysis buffer, and a portion was lysed in ATP assay buffer and centrifuged at 10,000 rpm for 15 min at 4°C to pellet insoluble materials. The supernatant was collected and ATP assay mixture was added in a 96-well plate, then the plate was incubated at room temperature for 30 minutes. The fluorometric signals at an excitation wavelength of 535 nm and emission wavelength of 587 nm was measured in SpectraMax M5 Multi-Mode Microplate Readers (Molecular Devices, Sunnyvale, CA). The concentration of ATP was calculated using ATP standard curve and expressed in nmol per mg protein. Protein concentrations in all brain samples were determined using BCA protein assay kit (Pierce, Rockford, IL).

### Histological Evaluation

At 2, 15 and 28 days after TBI, mice were deeply anesthetized and fixed by transcardial perfusion with phosphate-buffered saline (PBS) followed by perfusion and immersion in 4% paraformaldehyde. After the brains were removed and further fixed overnight, they were embedded in OCT compound (Sakura Finetek USA Inc., Torrance, CA), frozen in liquid nitrogen, cut into 15-µm-thick axial sections, and stained with hematoxylin and eosin (HE). Cavity area was measured by calculation for the percentage of the lesion area compared with the contralateral hemisphere area using Image J (NIH, Bethesda, MD).

### Statistical Analysis

Differences of neurological severity scores were evaluated by two-way repeated analysis of variance (ANOVA) with Bonferroni's *post hoc* test. In a two-dimensional coordinate system, the area-under-the-curve (AUC) data, which represent the time courses of NSS in the various groups of mice, were calculated using numerical integration [67]. Differences in the AUC between the untreated TBI and the laser-treated groups and between different laser-treated groups were compared for statistical significance using one way ANOVA.

Comparisons between the different groups in the other behavioral tests and the cavity measurement were performed using two-way repeated ANOVA with Tukey's *post hoc* test. Statistical analysis in the measurement of ATP contents was evaluated using one-way factorial ANOVA followed by Tukey's *post hoc* test. A value of *P*<0.05 was regarded as statistically significant.
